The article "Application of Isotope Tracer in Cross-Well Nanometre Tracer Testing" was retracted in 2023. Reasons: signs of a paper mill; suspected computer-generated content; unreliable results or conclusions; concerns about the data.

# Application of Isotope Tracer in Cross-Well Nanometre Tracer Testing

**DOI:** 10.1155/2022/6387030

**Published:** 2022-08-06

**Authors:** Yang Pang, Lin Zhao, Yushou Song, Guang Wei, Yehui Han, Qiang Wang

**Affiliations:** ^1^College of Nuclear Science and Technology of Harbin Engineering University, Harbin 150000, Heilongjiang, China; ^2^Heilongjiang Institute of Atomic Energy, Harbin 150000, Heilongjiang, China

## Abstract

In order to understand the dynamic monitoring characteristics and heterogeneity characteristics of injection production wells in the monitoring area and judge the reservoir connectivity, this study puts forward the application method of isotope nanometre tracer in interwell nanometre tracer testing. The trace material nanometre tracer interwell monitoring technology was applied to well block *J* in a basin. Through the analysis of the morphological characteristics of the nanometre tracer production curve and the quantitative interpretation of trace material tracer, combined with the analysis of the advancing speed of the water line at the front edge of the nanometre tracer and the distribution of injected water wells, the nanometre tracer connectivity, and advancing speed, the characteristics of seepage channels and heterogeneity of the well groups in the study area were defined. The research results show that 8 oil wells in the monitoring area are controlled by water injection well J1, the injection water inrush direction is generally north, the main channel of injection water is mainly high-permeability strip, and the heterogeneity contradiction between layers is strong. It is recommended to adopt mild water injection. *Conclusion*. This study found that the dynamic connectivity between oil and water wells in the monitoring area is good.

## 1. Introduction

Since the 1950s, oil field cross-well tracing technology has experienced great development in many countries in the world, from simple to deep, from qualitative interpretation to quantitative interpretation. The nanometre tracer selection, mineral construction, sampling analysis, and interpretation methods have been improved qualitatively [1]. The basic principle of interwell nanometre tracer test technology is to design the test scheme, select and prepare appropriate tracers by referring to the relevant dynamic and static data of the test well group, add tracers to the injection wells of the test well group, take samples and prepare samples in the surrounding production wells according to the established sampling system, conduct nanometre tracer analysis in the laboratory, and obtain the nanometre tracer content in the samples, as shown in Figure 1. In the early days, chemical tracers represented by inorganic salts, dyes, and halogenated hydrocarbons were used for cross-well tracer monitoring. Now, they are rarely used due to large amount, low detection sensitivity, and high cost. The isotope nanometre tracer represented by tritium water in the 1970s can be directly put into the well when used. It is easy to operate and can be detected with only a small amount of tracer. The price is also cheap. Therefore, it is still used as a commonly used nanometre tracer type [2]. However, as radioactive short-lived tracers are controlled by environmental protection, their application is limited, and it is necessary to cooperate with professional departments to complete relevant testing links. Therefore, a new type of tracers was proposed in the 1990s, mainly represented by trace elements (rare earth elements) and fluorescent tracers. However, the natural background of rare earth elements is high, and the detection sensitivity is limited, which also limits their wide application. Not only the selection of tracers is undergoing Longes but also some limitations and irrationalities in the process of theoretical research and mineral experiments are constantly being improved [3]. It mainly includes the progress of tracer detection technology, the improvement of testing technology, the development of a reservoir model and simulation technology, and the auxiliary verification of interpretation rationality. In recent years, with the increasing demand for enhancing ultimate oil recovery, the annual testing workload in China has reached more than 600 well groups. The testing process is also basically qualified, which can be safe and reliable. There is a standard testing system that can be implemented according to the actual situation. The cross-well tracing technology has a relatively complete system, which has played a role in guiding the oilfield development practice, understanding the formation characteristics of the reservoir, understanding the mechanism of tertiary oil recovery, and improving crude oil production and achieved good economic benefits [4].

The article "Application of Isotope Tracer in Cross-Well Nanometre Tracer Testing" was retracted in 2023. Reasons: signs of a paper mill; suspected computer-generated content; unreliable results or conclusions; concerns about the data.

## 2. Literature Review

Na, L. et al. developed a method to measure the fluid saturation of oil layer, which applies the chromatography theory. This method first injects the mixed liquid of the two tracers into the well and then produces in other production wells around. The two tracers will be separated due to different distribution coefficients. Therefore, it can be seen that the degree of their separation is related to the saturation of the remaining oil in the reservoir, which is a quantitative relationship. This is the method of using tracers to determine the saturation of the remaining oil in the reservoir. However, at that time, the application and development of this technology were hindered due to the inability to explain the tracer and the lack of a suitable tracer [5]. Zhu, X. and Ye, Y. invented a nanometre tracer by using water-soluble inorganic salts that are easy to identify, especially low-molecular alcohols and nitrates. This nanometre tracer fluid can improve the recovery of crude oil and can monitor the geological conditions formed between oil producing wells and water injection wells during oil production, as well as the flow relationship between them. Bacteria and some surface pollutants in oilfield water will decompose the tracer, so adding aromatic compounds can prevent the nanometre tracer from being degraded. The mass of aromatic compounds added is about 10∼2000 mg/l (50∼1500 mg/l is the best). The compounds include xylene, toluene, and benzene. These compounds are added to prevent microbial corrosion of the tracer [6]. Writer and C. P. S. T. determined the influence of mobile oil content on oil saturation calculation by analyzing the delay of distributive nanometre tracer data in chromatography [7]. Zhang, X. et al. studied the theoretical charts under different heterogeneity indexes and developed a method to study the heterogeneity of oil reservoirs by using them [8]. Li, Z. and Yan, X. also developed a method to explain reservoir heterogeneity, which also applies cross-well nanometre tracer data. Due to the different concentrations of tracers produced on the longitudinal profile, the tracers are sampled and analyzed at different depths underground, and indoor tests and simulation calculations are carried out to determine the formation parameters [9]. Zhong, K. et al. proposed that there are many kinds of tracers soluble in water that can be selected. In addition to the types containing tritium in the aqueous solution, radioactive 35 can also be selected to monitor the flowing liquid in the water injection well [10].

In order to understand the dynamic monitoring characteristics and heterogeneity characteristics of injection production wells in the monitoring area, judge the reservoir connectivity, and on this basis, systematically study the water breakthrough horizon, water breakthrough direction, and advancing speed of high water cut wells in the monitoring area, we should better understand the water drive law of injection production wells in the monitoring area and further describe the heterogeneity of well groups. Trace substance interwell nanometre tracer monitoring is carried out at the two horizons of Long 6_1_^1^ and Long 6_1_^2^ of well cluster 1 in the monitoring area.

## 3. Research Methods

### 3.1. Nanometre Tracer Screening and Dosage Design

#### 3.1.1. Nanometre Tracer Screening Principle

The fourth-generation cross-well nanometre tracer monitoring technology is adopted in this monitoring. Compared with the previous three generations, it is characterized by environmental protection of tracers, high detection accuracy of output concentration, no interference between tracers and formation fluids, and no adsorption effect. It can fully meet the requirements of this water drive tracer. There are more than 40 kinds of trace substances available [11]. On the premise of effective monitoring, the nanometre tracer screening shall try to achieve the minimum economic cost. According to the hydrogeological characteristics of well block *J*, the nanometre tracer type and dosage parameters of each layer shall be determined in combination with the nanometre tracer synthesis process. The type and amount of tracer are closely related to the type of reservoir horizon. Analyzing and processing the tracer fluid carried by oil well fluid production can obtain the information of fluid production in each interval. The concentration of a substance in the atmosphere or water after basically mixing is the background concentration of the substance. By analyzing the background natural quantities of 7 elements in the produced water of the oil well corresponding to the water injection well, it is found that the background concentrations of Yb and Er tracers are low. Yb and Er are preliminarily selected to inject tracers into well cluster J1, and output indication of tracers Yb and Er in long 6_1_^1^ and long 6_1_^2^ layers is simulated through experiments (Table 1) [12]. Based on the abovementioned data and the background concentration of the produced elements in the water injection well, it is finally determined that the tracers injected into well cluster J1 are Yb and Er, and layered injection is adopted.

The article "Application of Isotope Tracer in Cross-Well Nanometre Tracer Testing" was retracted in 2023. Reasons: signs of a paper mill; suspected computer-generated content; unreliable results or conclusions; concerns about the data.

#### 3.1.2. Nanometre Tracer Dosage and Sampling

The amount of tracer is determined by the heterogeneity, well spacing, thickness, porosity, water saturation, dilution outside the well pattern and between layers, formation surface adsorption, etc. Through years of research and a large number of field experiments, it is found that the “maximum dilution volume method” is a more suitable method for calculating the amount of trace substance nanometre tracer [13]. The volume of the monitoring layer and the minimum detection limit and sensitivity of the analytical method determine the amount of trace substance tracer. The calculation method is as follows:

(1) $$\begin{array}{c} V=\pi R^{2}H\phi S_{w}, \end{array}$$

(2) $$\begin{array}{c} A=\mu VM_{\text{DJ}}, \end{array}$$

where *V* is the maximum dilution volume, m ^3^;  *H* is the effective thickness of the sand body, m;  *R* is the average well spacing, m;  *ϕ* is the porosity calculated by the weighted average of the thickness of the oil layer in the monitoring layer, *f*;  *S*_*w*_ is the average water saturation of the monitoring layer, *f*; *A* is the amount of tracer, kg;  *μ* is the empirical guarantee coefficient, dimensionless; and *M*_DJ_ is the detection limit.

A total of 16 oil production wells are designed for sampling monitoring in this monitoring, and all of them can carry out normal sampling and testing. According to the geological conditions and development status of the monitoring area, the injection production well spacing of the monitoring well group ranges from 295.22 m to 790.93 m. The recent water cut Longe trend of the oil well is normal, and the injection water advance should be relatively uniform. The injection water may break through in a very short time. The initial sampling of the monitoring well is planned to be carried out 24 hours after the nanometre tracer injection and then once a day within 30 days to monitor the possibility of cracks or high-seepage channels in the formation; after 30 days of nanometre tracer injection, samples shall be taken every 2 days until the notice to stop sampling [14]. The sampling time range is from August 19, 2021, to November 18, 2021. The total sampling time span is 92 days. See Table 2 for nanometre tracer injection process parameters.

## 4. Result Analysis

### 4.1. Nanometre Tracer Application

#### 4.1.1. Well Cluster Conditions

The J1 well cluster is located in the middle of the 6_1_^1^ basin and is geologically located in the middle and west of the Northern Shaanxi Slope. The average effective thickness of a single well of the Triassic long 6_1_^1^ layer, the main oil layer in the monitoring area, is 13.5 m, and the effective permeability is  2.5 × 10^−3^*μ*m^2^; the average effective thickness of a single well in the long 6_1_^1^ formation is 16.8m, and the effective permeability is 2.78 × 10^−3^*μ*m^2^. The long 6 reservoir in well block *J* is a moderately strong heterogeneous reservoir [15]. Comparing the effective thickness, permeability, and other physical parameters of the long 6_1_ layer, the long 6_1_^2^ layer has longer facies, and the 6_1_^1^ layer has slightly better homogeneity, but the long 6_1_^2^ layer has more abundant seepage channels and more water can be seen in the development of fractures.

#### 4.1.2. Well Cluster Nanometre Tracer Connectivity Analysis

Comparing the production performance of the same nanometre tracer in the same layer with the table, when the nanometre tracer concentration curve has an obvious amplitude fluctuation trend, it is determined as the nanometre tracer well [16]. See Table 3 for the nanometre tracer production performance of each monitoring well in well block J1.

16 monitoring wells were successfully sampled from well cluster J1, and there were 8 obvious agent-seeing wells in total, with an agent-seeing ratio of 50%, indicating that these 8 wells were controlled by the water injection of water injection well J1, and the nanometre tracer seeing characteristics of Yb and Er were obvious. At present, the oil-water interwell performance of well cluster J1 in the monitoring area is good [17]. During the monitoring period, the nanometre tracer concentration production curve shows that there is a nanometre tracer production relationship between the J1 water injection well in the long 6_1_^1^ layer (element Yb) and the four oil wells (J2, J3, J4, and J5) with tracer; tracers are produced between long layer 6_1_^2^ (element Er) and the four monitored oil wells (J6, J7, J8, and J9). It indicates that water injection well J1 is connected with the abovementioned monitoring wells.

The article "Application of Isotope Tracer in Cross-Well Nanometre Tracer Testing" was retracted in 2023. Reasons: signs of a paper mill; suspected computer-generated content; unreliable results or conclusions; concerns about the data.

The shortest breakthrough time of nanometre tracer Yb is 7 days and the longest is 19 days, and the shortest duration of nanometre tracer Yb is 12 days and the longest is 35 days. In most cases, the middle of the wave peak is the peak position, and the peak value of nanometre tracer concentration fluctuates between (0.70∼1.86), indicating that the types of sweep channels of nanometre tracer Yb are relatively rich [18]. The shortest breakthrough time of tracer Er is 7 days, the longest is 47 days, the shortest is 9 days, and the longest is 22 days. The middle part of the wave peak is the peak position in most cases, and the peak value of tracer concentration fluctuates between (0.44∼0.70)  ng/mL, indicating that the types of sweep channels of tracer Er are relatively rich.

#### 4.1.3. Nanometre Tracer Propelling Speed Analysis

See Table 4 for oil well performance monitoring of well cluster J1. Based on the analysis of the nanometre tracer advancing speed of well cluster J1, the difference of agent breakthrough speed in a single well and different layers is large. The agent breakthrough speed of well J2 in layer 6_1_^1^ and well J6 in layer 6_1_^2^ is greater than 70 m/d, with an average agent breakthrough speed of 87.52 m/d. The agent breakthrough speed of the other six wells is generally less than 30 m/d, with an average agent breakthrough speed of 19.88 m/d [19]. There is no obvious linear relationship between the length of tracer breakthrough time and the well spacing of oil and water wells, and there is a negative correlation with the advancing speed of the front waterline, indicating that J2, J6, and J1 are well connected.

The article "Application of Isotope Tracer in Cross-Well Nanometre Tracer Testing" was retracted in 2023. Reasons: signs of a paper mill; suspected computer-generated content; unreliable results or conclusions; concerns about the data.

It can be seen from Table 4 that the nanometre tracer has a relatively single direction to the north as a whole and abundant nanometre tracer forms, and there is no obvious linear relationship between the injection water distribution and the advance speed of the front waterline. The average advancing speed of the waterline front of long layer 6_1_^1^ is 34.89 m/d, while the average advancing speed of the waterline front of long layer 6_1_^2^ is 35.89 m/d, and there is no significant difference [20]. The advancing speed and direction of the water front of well J1 can be calculated according to the distance between oil and water wells and the breakthrough time of tracer. The nanometre tracer injected into layer 6_1_^1^ has a shorter breakthrough time, and the water drive speed from well J1 to well J2 and well J6 is significantly faster than that of other wells in the same layer [21]. It can be inferred that the obvious difference of water drive speed between J1 well and J2 well and J6 well and other agent seeing directions is related to the water injection history of the well group. There may be a high seepage channel formed by long-time water injection scouring in the J2 well and J6 well, and the heterogeneity between oil and water wells is strong.

#### 4.1.4. Analysis of Seepage Channel Characteristics

The consistency between the original nanometre tracer concentration curve and the fitted curve is related to the difference between the distribution of formation parameters in the model and the actual situation. The higher the consistency between the original nanometre tracer concentration curve and the fitted concentration curve, the smaller the difference between the physical model and the actual situation of the formation. Generally, the peak concentration of nanometre tracer production curve fluctuates with the thickness and permeability difference of each injection and production well in the monitoring well area. Microfractures or high-permeability bands are the key for the nanometre tracer to break through the oil wells in the monitoring area. When the nanometre tracer enters these areas with the injected water, the peak concentration will appear. Generally, the number of peaks is the number of high-permeability bands or microcracks [22]. The characteristics of injected water along fractures or high-permeability bands are shown in the tracer concentration curve as follows: the trace of tracer production is clear, there are many peaks with clear peak shape, the peak value is prominent, the duration is short, and the concentration curve is relatively smooth. See Figure 2 for the nanometre tracer Yb production concentration curve of well J5. The consistency between the calculated formation parameters and the actual formation conditions is positively correlated with the consistency between the original curve and the fitting curve.

The article "Application of Isotope Tracer in Cross-Well Nanometre Tracer Testing" was retracted in 2023. Reasons: signs of a paper mill; suspected computer-generated content; unreliable results or conclusions; concerns about the data.

#### 4.1.5. Heterogeneity Analysis

Because the nanometre tracer has different breakthrough time on oil wells with different injection production well spacing, the water front velocity of each well group is calculated and analyzed. By comparing the nanometre tracer monitoring well groups of long 6_1_^1^ and long 6_1_^2^ horizons in well block *J*, it is found that the minimum waterline front advance speed is 12.83 m/d, the maximum waterline front advance speed is 100.45 m/d, and the median value is 36.74 m/d. It can be seen that the water drive speed in the well group varies greatly with the breakthrough time of each associated oil well [23]. Reservoir heterogeneity can be divided into interlayer heterogeneity, intralayer heterogeneity, and plane heterogeneity. According to the heterogeneity evaluation standard and the layered evaluation results of water drive velocity heterogeneity, there is no obvious difference in interlayer water drive velocity of well cluster J1, and the interlayer heterogeneity is weak. The evaluation result of water drive velocity heterogeneity in the long layer is medium, while that in long layer 6_1_^2^ is strong, and the overall evaluation result is medium to strong [24]. According to the evaluation and analysis in Table 5, the permeability difference of the main channel in the well cluster is obvious, corresponding to the fast water drive speed between injection and production wells, strong heterogeneity between layers, and prominent heterogeneity contradiction within layers.

## 5. Conclusion

Trace material tracing monitoring technology can effectively judge the corresponding relationship between oil and water wells within and between layers. Among the 16 sampling wells monitored by the trace substance tracer, 8 wells were found agent, and the agent discovery rate was 50%. Therefore, the dynamic connectivity between oil and water wells in the monitoring area was good. The research shows that the J2 well in the long 6_1_^1^ layer and the J8 well in the long 6_1_^2^ layer are the main flow channels of the well group, and the injection water ratio is 45.05% and 20.31%, respectively, which is significantly higher than that of other injection wells in the same layer. There is a great difference in the advancing speed of water front between injection and production wells in each monitoring well section, and there is a strong plane heterogeneity contradiction between layers and within layers. The oilfield is a low-permeability reservoir. In order to avoid severe fluctuations in reservoir physical properties caused by strong production and injection, which may lead to difficulties in later development of the oilfield or even serious consequences, it is recommended to adopt mild water injection.

The article "Application of Isotope Tracer in Cross-Well Nanometre Tracer Testing" was retracted in 2023. Reasons: signs of a paper mill; suspected computer-generated content; unreliable results or conclusions; concerns about the data.

## Figures and Tables

**Figure 1:** Cross-well nanometre tracer test.

**Figure 2:** Tracer Yb production concentration curve of well J5.

**Table 1:** Nanometre tracer type selection of well cluster J1.

Simulated horizon	Tracer primary screening	Relative dosage (%)	Tracer indication	Tracer selection	Corresponding well
Long 6_1_^1^	Yb	25	Strong	Yb	J2, J3, J4, and J5
	Er	25	Weak		

Long 6_1_^2^	Yb	25	Weak	Er	J6, J7, J8, and J9
	Er	25	Strong		

**Table 2:** Nanometre tracer injection process parameters.

Well cluster	Injection mode	Injection horizon	Tracer type	Tracer (kg)	Solution concentration *wt* (%)	Water consumption(m^3^)
J1	Concentric double-pipe separate injection	Long 6_1_^1^ (outer pipe)	Yb	33	1	3.5
		Long 6_1_^2^ (inner pipe)	Er	26	1	3.0

**Table 3:** Tracer production performance of tracer wells.

See agent well	Well spacing (m)	Breakthrough date	Tracer concentration (ng*·*mL ^−1^)	Peak date	Tracer concentration (ng · mL ^−1^)	End date	Duration (d)
J2	522.12	2021-08-25	0.15	2021-08-26	0.78	2021-09-28	35
				2021-09-09	0.70		
J3	300.78	2021-09-06	0.13	2021-09-09	0.88	2021-09-17	12
J4	309.28	2021-09-03	0.14	2021-09-05	0.78	2021-09-17	15
J5	387.62	2021-08-31	0.17	2021-09-16	1.86	2021-09-30	31
J6	703.15	2021-08-25	0.01	2021-08-27	0.44	2021-09-02	9
J7	295.22	2021-08-30	0.18	2021-09-01	0.65	2021-09-14	16
J8	513.25	2021-09-27	0.09	2021-09-28	0.70	2021-10-18	22
				2021-10-05	0.54		
J9	790.93	2021-10-14	0.03	2021-10-08	0.44	2021-10-14	11

**Table 4:** Dynamic monitoring of well cluster J1.

Tracer	Corresponding well	Distance between oil and water wells (m)	Tracer breakthrough time (d)	Leading edge waterline propulsion speed (m · d^−1^)	Injection water ratio (%)	Injection water distribution (m^3^ · d^−1^)	Actual water production (m^3^ · d^−1^)
Yb	J2	522.12	7	74.59	45.05	5.86	2.80
	J3	300.78	19	15.83	6.38	0.83	1.00
	J4	309.28	16	19.33	7.15	0.93	0.76
	J5	387.62	13	29.82	8.21	1.07	0.29

Er	J6	703.15	7	100.45	20.20	0.34	0.35
	J7	295.22	12	24.26	15.64	2.66	1.79
	J8	513.25	40	12.83	20.31	3.45	1.31
	J9	790.93	47	16.48	6.90	1.17	0.98

**Table 5:** Tracer production channel thickness coefficient of injection production wells.

Thickness (cm)			Grade difference	Inrush coefficient	Coefficient of variation	Evaluation results
Maximum	Minimum value	Average value				
7.58	0.21	2.71	36.10	2.80	0.78	Secondary

The article "Application of Isotope Tracer in Cross-Well Nanometre Tracer Testing" was retracted in 2023. Reasons: signs of a paper mill; suspected computer-generated content; unreliable results or conclusions; concerns about the data.

## Data Availability

The data used to support the findings of this study are available from the corresponding author upon request.
